# Finite Element Simulations of Mechanical Behaviour of Endothelial Cells

**DOI:** 10.1155/2021/8847372

**Published:** 2021-02-16

**Authors:** Veera Venkata Satya Varaprasad Jakka, Jiri Bursa

**Affiliations:** Institute of Solid Mechanics, Mechatronics and Biomechanics (ISMMB), Faculty of Mechanical Engineering (FME), Brno University of Technology (BUT), Technicka 2896/2, 61669 Brno, Czech Republic

## Abstract

Biomechanical models based on the finite element method have already shown their potential in the simulation of the mechanical behaviour of cells. For instance, development of atherosclerosis is accelerated by damage of the endothelium, a monolayer of endothelial cells on the inner surface of arteries. Finite element models enable us to investigate mechanical factors not only at the level of the arterial wall but also at the level of individual cells. To achieve this, several finite element models of endothelial cells with different shapes are presented in this paper. Implementing the recently proposed bendotensegrity concept, these models consider the flexural behaviour of microtubules and incorporate also waviness of intermediate filaments. The suspended and adherent cell models are validated by comparison of their simulated force-deformation curves with experiments from the literature. The flat and dome cell models, mimicking natural cell shapes inside the endothelial layer, are then used to simulate their response in compression and shear which represent typical loads in a vascular wall. The models enable us to analyse the role of individual cytoskeletal components in the mechanical responses, as well as to quantify the nucleus deformation which is hypothesized to be the quantity decisive for mechanotransduction.

## 1. Introduction

Atherosclerosis is a leading cause of morbidity and mortality in the developed world. It is characterized by progressive narrowing and hardening of arteries which lead to ischemia of the heart, brain, or extremities and may cause infarction or stroke [1]. To elucidate the atherogenesis, it is important to understand the cellular responses to mechanical stimuli exerted on endothelial cells from their haemodynamic environment or artery deformation.

The endothelium is a monolayer of endothelial cells that line inner walls of arteries, hence providing an interface between the flowing blood and the artery wall [2] and playing a key role in the pathobiology of atherosclerosis [3]. The endothelial cells are of flat hexagonal shape [4, 5] elongated in the blood flow direction [6].

Living cells are highly complex structures consisting of a large number of distinct structural components such as the cytosol, cell membrane (CM), cytoskeleton, nucleus, and other organelles. The cytoskeletal network is composed of three types of components, namely, actin filaments (AFs), microtubules (MTs), and intermediate filaments (IFs), which are spread throughout the cytoplasm and interlinked to each other, to the nucleus, and to the CM [7]. Their structural arrangement is decisive for the response of the cytoskeleton to mechanical stimuli and for the stiffness of the whole cell. The prestress in AFs is balanced mainly by MTs but partly also by continuum parts and the extracellular matrix, to which the cell is tethered [8].

In the past few decades, the development of microrheological techniques [9] has made quantitative mechanical measurements of single living cells feasible. For our research, the following testing methods are most relevant: microplate stretcher [10], microplate manipulation [11, 12], and atomic force microscopy (AFM) [13]. There are other more recent techniques which can reveal the mechanical characteristics of cells such as a microfluidic device [14], dissipative particle dynamics [15], or micropipette aspiration [16, 17].

Some recent models of cell mechanics consider their structure to include the cytoskeleton, e.g., the multistructural model [18], the spring network cell model [19], and the granular cell model [20]. Other studies of active approaches incorporate the cell's inherent active nature in computational modelling such as the bio-chemo-mechanical model [21], the dynamic stochastic model [22], and the kinematic model [23]. Although these models are equipped with formulations to explain both passive and active responses of cells, they do not elucidate the contribution of cytoskeletal components. This is feasible with tensegrity-based finite element (FE) models consisting of both tension- and compression-bearing elements [24] which show a self-stabilizing effect [25].

In order to interpret the relation between the biological response of living cells and mechanical stresses, tensegrity models are predominantly suitable for cytoskeletal structures of living cells [26]. However, in cytoskeletal tensegrity models presented in the literature, the MTs appear too stiff because they do not account for the flexural behaviour of MTs [27]. In order to overcome this problem, the most sophisticated hybrid model has been recently created using the bendotensegrity concept [28] for modelling smooth muscle cells [29]. This concept was adopted also in this study, and the model was modified to represent specific features of endothelial cells and the role of individual cytoskeletal components in their mechanical response.

## 2. Materials and Methods

For the simulation of mechanical tests of an endothelial cell, FE models with different shapes were created using the commercial software ANSYS (ANSYS Inc., USA). The hybrid modelling approach is similar to the model of the vascular smooth muscle cell in [30], where the cytoplasm, nucleus, and CM are modelled with continuum elements while the individual cytoskeletal components are modelled as discrete (unidimensional) elements. This approach enables us to study the mechanical role of individual cytoskeletal components in cellular mechanical response as well as the propagation of mechanical stimuli throughout the cell, including quantification of nucleus deformation under different types of loads. Both the cytoplasm and nucleus were modelled with eight-node hexahedral isoparametric elements. A thin flexible layer circumscribing the cytoplasm referred to as CM was modelled with four-node quadrilateral shell elements on the outer surface of the cytoplasm, with no bending stiffness and a thickness of 0.01 *μ*m [31], coupled with the 3D elements through nodal displacements only, thus leaving nodal rotations of the shell free. The cytoskeleton (with the same topology in all the models as described below) was inscribed inside the continuous part thus creating the hybrid model.

Three different mechanical tests were simulated to validate the proposed model: tensile and compression tests of a suspended (spherical) cell with micropipettes and microplates, respectively, and a compression test of the cell adhered to a substrate which thus had the shape of a truncated sphere. The model of the endothelial cell in its typical flat shape in the endothelium layer cannot be validated due to lack of experimental data. Therefore, this flat model was created on the basis of the above validated models, keeping their topology and volume; then, it was used for the simulation of compression and shear of the endothelium cell in its natural shape. Based on its physiological dimensions and shape, the cell was modelled as a very short flat regular hexagonal prism [4, 32] with a thickness of 0.5 *μ*m [4, 33, 34] as shown in Figure 1(b). In order to investigate an even more physiological shape, the flat model was then modified into a dome with the cell being 20% higher at the centre than at the edges; this nonuniform height corresponds better to the physiological endothelial shape [14, 35].

The cytoskeletal arrangement is decisive for the mechanical and possibly also for the biochemical response of living cells [8, 36, 37]. The cytoskeleton in our model comprises 12 beam elements (representing the MTs which are curved, all connected in the centrosome, and capable of bearing flexion and tension or compression), 36 prestressed truss elements (representing the AFs and bearing tension only), and 24 truss elements representing the IFs. To mimic their waviness, the IFs have a prestrain of 20 percent to resist tensile loads only under larger elongations [38–40]. In contrast, the experimentally measured prestrain of 24% [41, 42] was always assigned to AFs in the first load step to generate their prestress (initial force without load) essential for the cell shape stability.

The MTs of unequal lengths originate from the centrosome, represented by a node located near the nucleus. They emanate outward through the cytoplasm till the cortex where they interact with other cytoskeletal filaments at focal adhesions (FAs). Due to the different nature of truss and beam elements, the rotational degrees of freedom of beams remain free here, and no other contacts (and consequently no friction) are assumed between the MTs and the continuum elements representing the cytoplasm. The authors believe that this behaviour of MTs (but also of AFs and IFs) corresponds to the fluid nature of the cytosol and to the character of the FAs. Every FA is connected to the centrosome with only one MT, and it is ensured that they do not penetrate the nucleus.

IFs are scattered throughout the intracellular space, connecting the FAs to the nucleus and creating a dense network in the perinuclear region that stabilizes the nucleus at the cell centre [39]. For better transmission of mechanical stimuli to the nucleus and its stabilization at the centre of the cell, each FA was connected to the nucleus via at least two IFs. To mimic their real structural arrangement, they were modelled tangentially to the nucleus, thus creating a dense network in the perinuclear region.

For the flat cell model, thin AFs were stretched between each pair of 12 nodes of the hexagonal prism, except for those which would penetrate the nucleus. The same arrangement was used in the dome and spherical model. In the adherent cell, actin is arranged in thick longitudinal bundles (ABs), the arrangement of which is described in detail in Section 2.3.

### 2.1. Material Properties

Although the cytoplasm behaves as a liquid rather than as a solid, the shear stresses induced in it during (static, i.e. relatively slow) mechanical tests are negligible. Thus, a very low compressibility represents its basic feature, which can be modelled using the Neo-Hookean model given by the following formula for its strain energy density *W*:

(1) $$\begin{array}{c} W=\frac{G}{2}\left(\bar{I_{1}}-3\right)+\frac{1}{d}{\left(J-1\right)}^{2}, \end{array}$$

where *G*(Pa) is the initial shear modulus, *d*(Pa^−1^) is the compressibility parameter, *J* is the 3rd determinant of the deformation gradient tensor, and $\bar{I_{1}}$ is the 1st invariant of the isovolumic part of the right Cauchy-Green deformation tensor. To keep the negligible shear stresses, the shear modulus was set very low (170 Pa). For the cell membrane, the material parameters were calculated from the known elastic constants as follows:

(2) $$\begin{array}{c} G=\frac{E}{2\left(1+\upsilon \right)},\\ K=\frac{E}{3\left(1-2\upsilon \right)}=\frac{2}{d}, \end{array}$$

where *E*(Pa) is Young's modulus, *υ*(−) is Poisson's ratio, and *K*(Pa) is initial bulk modulus.

For the cytoskeleton, we use the following linear elastic model:

(3) $$\begin{array}{c} \varepsilon =\frac{\sigma }{E}+\varepsilon_{0}, \end{array}$$

where*σ*(Pa) is engineering stress, *ε*(−) is engineering strain, and *ε*_0_(−) is applied prestrain which is negative for AFs and positive for IFs. All the parameters are summarized in Table 1 and Table 2 with the literature they are based on. The nonrealistic values of Poisson's ratio for cytoskeletal elements (0.3) are taken from the literature [18, 30, 43, 44] and have no impact on the results because they are represented as a 1D element.

### 2.2. FE Model for Suspended (Spherical) Endothelial Cell

In order to validate the simulated mechanical response of the endothelial cell, we rearranged the flat endothelial cell model into a spherical shape occurring in experiments [47]. For this purpose, we assumed the same volume of the cell, which gave us two concentric spheres representing the cytoplasm and the nucleus with diameters of 7.4 *μ*m and 3.0 *μ*m, respectively. The cytoskeletal arrangement of the spherical cell is shown in Figure 2(a).

#### 2.2.1. Boundary Conditions for Compression

Compression of the cell was simulated for comparison with the experimental cell response in a compression test done with microplates [47]. To avoid difficulties related to the contact between the cell and the microplates (which are supposedly rigid), the cell model was fixed in its central node in all directions and vertical displacements were prescribed on both top and bottom sides to flatten the area being in contact with the microplates, and to achieve 50% shortening of the cell vertical dimension (see Figure 2(b)).

#### 2.2.2. Boundary Conditions for Tension

The tensile test of a suspended cell was simulated in several steps for comparison with the cell response during stretching with rigid micropipettes [49]. With AFs being prestressed in the first load step, a bonded contact between the spherical cell and the faces of both micropipettes was established in the second load step by compressing the cell by approximately 20% (see Figure 3(b)). In the third load step, the cell was elongated to achieve zero reaction forces in the micropipettes; this unloaded state defines the initial length of the cell for calculation of its global relative deformation (strain) evaluated in percentage similarly to the experiments. In the final load step, uniform displacement was applied to the nodes of the top and bottom surfaces to achieve 50% elongation of the model (see Figure 3(c)).

### 2.3. FE Model of Adherent Endothelial Cell

The model with an axisymmetric truncated spherical geometry possessed a maximum diameter of 20 microns and a maximum height of 8 microns, with the nucleus having a flat ellipsoidal shape, and the centre placed in half height of the model; its major and minor (height) axes are 8 microns and 4 microns, respectively, based on experimental observations [47, 50].

To consider a different structural arrangement of the adherent cell [30], thick actin bundles (ABs) were incorporated in the model instead of AFs (with the same prestrain); they were observed at the cell periphery running almost uniformly in the longitudinal direction [18, 41]. Moreover, a thin layer of actin-gel referred to as actin cortex (AC) was added to the shell elements on the cell model surface to represent both CM and the subcortical network of AFs. The experimentally measured thickness of the cortical layer of 0.2 *μ*m was chosen for our model [51, 52], being 20 times higher than the cell membrane itself; this value is consistent with another study on endothelial cells [50]. The arrangement of the cytoskeletal components of the adherent cell model (ABs, MTs, and IFs) is shown in Figure 4.

#### 2.3.1. Boundary Conditions of Adherent Cell in Compression

To validate a model with a modified geometry and structure, simulation of a compression test of an adherent endothelial cell done with microplates was performed with boundary conditions mimicking the experimental approach [47]. After application of the prestress to the ABs, the cell was fixed at the bottom surface to mimic the (rigid) substrate and compressed vertically on the top side by application of vertical displacements to the nodes coming gradually into contact with the upper rigid microplate; these displacements were calculated in order to flatten the contact area and to achieve the total 50% deformation of the cell (see Figure 5). The reaction force was evaluated as the sum of forces at nodes of the top side of the cell.

### 2.4. Flat and Dome FE Models for Endothelial Cell

The hexagonal shape of the flat cell model (with an edge length of 12.5 microns and a thickness of 0.5 microns) is typical for cells creating an endothelial layer. The nucleus is ellipsoidal with a major (horizontal) axis of 9 microns and a minor axis (height) of 0.4 microns, located again symmetrically on top view and with a spacing of 0.05 microns between the bottom surfaces of the cell and nucleus. The arrangement of its individual cytoskeleton components is shown in Figures 1(a) and 1(b). With this model, two typical types of physiological load were simulated, namely, compression (being equivalent to biaxial tension in the arterial wall) and shear, induced by viscous forces from the blood flow. The dome model was then created by increasing the height by 20% in the central region of the cell to mimic better the real shape in the vascular endothelium (see Figure 1(c)). Then, it was used to investigate the shear response and to assess the impact of nonuniform cell thickness on shear response in the physiological hexagonal cell shape.

#### 2.4.1. Boundary Conditions

To mimic the compression experiment [47], the endothelial cell model was compressed in the thickness direction (symmetrically on top and on the bottom side) to achieve a 50% reduction of the cell height. The resulting reaction force was evaluated as a sum of the reaction forces in nodes either on top or on the bottom surface.

The shear load of the flat endothelial cell model was simulated in two steps. In the first step, all the nodes of the bottom hexagonal face were fixed in all directions and the cell was loaded in all the surface nodes on the top side by prescribed displacements reaching 15% of the cell height in *x*-direction. The resulting reaction forces where then applied in a new simulation at all the nodes on the top side of the cell model, and the same load was applied also on the dome model. In this way, the force-controlled load was applied, corresponding to real shear forces induced by the blood flow and being the same at both models for their direct comparison.

### 2.5. FE Mesh Density

For all the solved models, the meshes counted between 5 and 18 k elements; their sufficient density was confirmed as follows. When the mesh size was reduced to a half, the number of elements increased by a factor of approximately 8. With this denser mesh, the calculated maximum strains in the nucleus as well as the other quantities related to the continuum part increased by 3-4% while the stresses in beam elements (MTs) changed even less and the link elements (AFs, ABs, and IFs) were insensitive to the number of elements.

## 3. Results

With the exception of the shear load, the symmetric geometrical shape of the model and the arrangement of the cytoskeleton resulted in a nearly isotropic behaviour of the model without a preferred orientation.

### 3.1. Results for Suspended Cell Compression

The force-deformation curve calculated from the compression test simulation is in good agreement with the experimental curves in normalized form obtained from the compression tests of cultured endothelial cells [47, 53] and also shows a similar strain stiffening (see Figure 6). This strain stiffening occurring with all the investigated shapes of the cell (see also Figures 7 and 8) is reached by mimicking the cytoskeleton with tensegrity structures; they show strain stiffening as their basic feature even if made of linear elastic materials. The cell diameter in the experiments differs from our model; thus, for comparison, the experimental reaction force *F* was transformed into *F*_*N*_ by normalization to the same diameter.

(4) $$\begin{array}{c} F_{N}=F{\left[\frac{D}{D_{\exp}}\right]}^{2}, \end{array}$$

where *D* is the diameter of the model, and *D*_exp_ is the cell diameter in the experiment.

The logic of normalization is based on proportionality between the cell cross-section area and the resulting force under the same stress.

The MTs in the central region being perpendicular to the direction of loading are straightened and bear much higher tensile forces while the others remain bended (see Figure 9(c)). Also, the AFs reoriented perpendicularly to the loading direction resist high tensile stresses as shown in Figure 9(a), and their number increased with cell compression. In contrast, the IFs reoriented perpendicularly to the direction of compression are only slightly uncoiled from their initial waviness, and exhibit very lower positive stresses presented in Figure 9(b).

The nucleus appears elongated in the transversal plane perpendicular to the loading direction, analogous to that observed in experiments [47]. The maximum first principal strain in the nucleus (see Figure 9(d)) was chosen as the quantitative characterization of nucleus deformation which is hypothesized to be decisive for transducing mechanical signals into changes in gene expression [54, 55].

### 3.2. Results for Suspended Cell Tension

The force-elongation curve calculated from the tensile test simulation is in good agreement with the experimental response, as illustrated in Figure 7 where the experimental results are also in their normalized form as described in Section 3.1.

The stiffness of the hybrid model of a suspended cell in tension was evaluated as secant modulus *σ*/*ε* of the resulting curve recalculated into conventional stress (*σ*) and conventional strain (*ε*). The conventional stress is given as:

(5) $$\begin{array}{c} \sigma =\frac{f}{a}, \end{array}$$

where *f* = 0.0765 *μ*N is the reaction force at maximum deformation of the cell, and *a* = 42.9866 *μ*m^2^ is the (maximal undeformed) cross-sectional area of the cell. With reference to Figure 7, the modulus of 3.17 kPa calculated for the FE model (*D* = 7.4 *μ*m) is in concordance with the modulus of 2.6 ± 0.7 kPa calculated for the experiments [49]. The cell stiffness increases with load in accordance with [19, 56], and the proposed model can predict the contribution of specific cytoskeletal components to the cell stiffness. The randomly oriented AFs tend to be aligned in the loading direction and to show high stresses as represented in Figure 10(a), which increases the overall reaction force of the cell. Also some MTs are merely straightened out while some others remain bended as shown in Figure 10(c). IFs aligned in the direction of the load are straightened and exhibit significant stresses while zero stress occurs in the others which remain wavy (see Figure 10(b)). The maximum first principal strain in the nucleus (see Figure 10(d)) is also presented as the quantitative characterization of nucleus deformation.

### 3.3. Results for Adherent Cell Compression

The simulated force-deformation curve is in good agreement with the experimental responses obtained from the compression test of endothelial cells cultured on a rigid substrate [47], including their strain stiffening, as represented in Figure 8. The distribution of the first and third principal strains in the nucleus is represented in Figure 11. The reason for showing also the third principal strain is that in compression its absolute value is higher than that of the first principal strain, and thus it might be decisive for mechanotransduction under these conditions.

### 3.4. Results for Compression of Flat Cell Model

The stiffness of the flat model (see Figure 8) is several times higher than that of the adherent model or of the spread cells obtained experimentally [47]. The reason is the different shape of the model (very short hexagonal prism) when the shape cannot change so much and the impact of volume incompressibility is much higher. Distribution of the first and third principal strains in the nucleus of the flat endothelial cell model under compression is shown in Figure 12.

### 3.5. Results for Shear of Flat Cell Model

Total reaction force calculated as the sum of reactions in nodes of the top hexagonal plane was *F*_*S*_ = 759 pN. As the area of the regular hexagon is *A*_*H*_ = 405.95 *μ*m^2^ (with a side length of 12.5 *μ*m), the resultant shear stress is *τ* = *F*_*S*_/*A*_*H*_ = 1.87 Pa, which is within the physiological range of wall shear stress in arteries. The same results were obtained with the corresponding force-controlled load of the model. The maximum first principal strain in the nucleus was about 0.039, and its distribution is presented in Figure 13(a). When the same forces were applied in the nodes of the top surface of the dome model, the maximum first principal strain in the nucleus was about 0.029 (see Figure 13(b)), i.e., some 26% lower. This difference shows that the local differences in thickness [14, 35] captured by the dome model may be significant, and the dome shape of the endothelial cell model should be preferred to its flat shape.

The maximum shear strain (in *xy* plane in which the shear stress is acting) within the whole cell occurs in the cytoplasm above the nucleus; it is 0.50 for the flat model and 0.40 for the dome model (see Figure 14). In contrast, the nucleus undergoes much lower strains as it is 10 times stiffer than the cytoplasm and the shear deformation is concentrated in the cytoplasm above and below the nucleus. Evidently, the transmission of strain to the nucleus is much lower in shear than under the other loading conditions, probably due to a lower role of cytoplasm incompressibility in shear.

### 3.6. Contribution of Cytoskeleton to Cell Stiffness

The role of each cytoskeletal component in cell stiffness was investigated via removal of this component from the hybrid model as illustrated in Figures 15 and 16 comparing the stiffness of the modified models, i.e., the total reaction force under the same (maximum) deformation. The results in Figure 15(a) show that the stiffness of the spherical model in compression decreases by some 32% when all the cytoskeleton components are removed; the contribution of AFs to the stiffness appears to be the highest: compared to the reaction force of the hybrid model, removal of AFs reduced the reaction force of the cell model by 20%. This rather contraintuitive result relates to volume incompressibility of the cytoplasm and a consequent increase in lateral dimensions of the cell under compression.

In simulations of the tensile test of the spherical model, the maximum reaction force of the cell model without a cytoskeleton was 66% lower than that for the hybrid model (see Figure 15(b)), and both AFs and MTs played a vital role in this decrease.

Investigation done with adherent and flat cell models under compression brought results qualitatively similar to those with the spherical model under compression, as illustrated in Figure 16.

## 4. Discussion

A new hybrid FE model of endothelial cells was exploited for simulations of mechanical responses of cells with different shapes and under different types of loads. It was validated by comparison of the calculated responses with experiments done with suspended endothelial cells in tension and compression, and with a compression test of an adherent cell. The same concept, topology, structure arrangement, and material properties were used in the flat and dome models of the hexagonal endothelial cell, which correspond more or less to its common shape within the vascular endothelium layer. These models were used to simulate the cell response under compression and shear, representing types of loads typical for “*in vivo*” endothelial cells. While shear load is induced directly by the blood flow as captured by the presented models, compression (in radial direction) represents an approximate equivalent of biaxial tension. However, this holds accurately only for homogeneous, isotropic, and incompressible materials; thus, biaxial tension (in circumferential and axial directions) should be preferred in the future, corresponding to the real load of the endothelial cells in the arterial wall.

In addition to the realistic simulation of experiments, the proposed model can predict stress/strain distribution within the specific cell components under different types of loads, as well as the impact of individual cytoskeletal components on the cell response. Thus, it surpasses not only all continuum models of cells [18–23] but also the tensegrity models envisioning the AFs as tension supporting cables and MTs as compression supporting struts [8]. Although these models explain successfully several observations in cell mechanics [43], they neither take into account the influence of flexural behaviour of MTs nor predict the impact of individual cytoskeletal components nor mimic the load transmission onto the nucleus. Moreover, the excessive compression stiffness of the struts introduces nonrealistic artefacts in mechanical responses, as shown in [27, 57]. The cell model based on the bendotensegrity concept was proposed in [30] for smooth vascular cells, but to the best knowledge of the authors, such models have not been used for endothelial cells till now. The published models of endothelial cells are mostly much simpler [4], and the role of the cytoskeleton is seldom investigated in existing literature. The recent study in cell mechanics simulated the mechanical behaviour of a cell with an oversimplified tensegrity structure, and the role of individual filaments was not accessed [44, 58]. However, there are studies analysing the role of the cytoskeleton in cell mechanics [30, 59]. Moreover, some published FE models on cell mechanics deal with the degradation of the cytoskeleton using more simplified cytoskeletal arrangements [60].

Among the cell components, the nucleus plays a vital role in mechanotransduction; thus, its deformation, described locally by strain tensor, may be decisive in the initiation of the cell's biochemical response to mechanical load. Within the strain tensor, we hypothesize that the component with the highest absolute value (either first principal strain *ε*_1_ or third principal strain *ε*_3_ if its absolute value exceeds *ε*_1_) is decisive. Therefore, these strain components are preferentially evaluated. Naturally, for confirmation of this hypothesis, challenging comprehensive mechanical-biological studies are needed.

In contrast to stress, more frequently used in mechanics, the advantage of our choice of strain as the decisive quantity is its much lower dependence on material properties. Constitutive models of materials represent an important limitation of any computational cell model due to lack and large dispersion of experimental data concerning individual cell components, and the consequent simplification of their responses via Hookean (linear elastic) or neo-Hookean (simplest hyperelastic) models.

Our model gave maximal *ε*_1_ values of 0.18 and 0.22 under 50% global deformation in compression and tension of a suspended cell, respectively, 0.19 in an adherent endothelial cell under 50% compression, 0.25 in a flat endothelial cell under 50% compression, and 0.039 and 0.029 in flat and domed endothelial cells under a physiological magnitude shear load, respectively. All these values are logarithmic (natural) strains. It is well established that cells respond to mechanical stimuli in a variety of ways that range from changes in cell morphology to activation of biochemical responses [61], which may affect the cell phenotype. Based on the proposed model, the amount of nucleus deformation could enable the researcher to compare mechanobiological responses under different mechanical stimuli.

The simulations realized with the created models give mechanical responses in accordance with experiments under different types of loads and enable a deeper analysis of the role of individual cytoskeletal components in cell stiffness. It was shown that, in any shape of the cell and under any type of load, the prestressed AFs are most significant for the cell stiffness; for instance, simulations of tension and compression tests with a spherical (suspended) cell model demonstrated that removal of AFs reduced the cell stiffness by approximately 23% and 20%, respectively. This modification of the model corresponds to cell treatment with cytochalasin D that results in disruption of not only the deep actin fibres but also of the actin meshwork beneath the CM [11]. The role of the other components is less pronounced; the initially wavy IFs contribute to cell stiffening with increasing load due to their reorientation and straightening, thus contributing to the nonlinear cell response. A similar effect occurs with the bended MTs when some of them become straight under load. This is the case specifically under high tension (see Figure 15(b)). Although the proposed models have advantages over the previous models, they have more limitations than those mentioned above. The structural arrangement of cytoskeletal components does not capture their true complexity and dynamic behaviour as observed in living cells. These models also do not take into consideration the viscoelastic nature of cells. Thus, they cannot predict very fast responses of the cell in which the viscoelastic nature of the cytoplasm (and possibly also of other components) becomes significant. Due to their passive nature, none of these models can capture active responses of the cell such as remodelling of AFs and MTs exhibited with respect to mechanical loading when the cytoskeletal fibres undergo polymerisation and depolymerisation. However, this remodelling occurs in time periods much longer than the duration of the considered experiments; thus, they cannot be captured either by the experimental responses.

As concerns the cell shape, within the arterial wall the endothelial cells are elongated in the direction of blood flow while we have considered a regular hexagon for idealization. However, the differences cannot be pronounced and the shape can be easily changed if the presented flat and dome models are applied in the future for investigation of adhesion between the cells and of possible disruption of the endothelial monolayer.

### 4.1. Limitations of the Model

Although our model considers the basic nonlinear feature of filaments, i.e., prestress in AFs and prestrain (waviness) of IFs, it cannot consider their strain stiffening [62] due to software limitations. However, within the range of some 10% strain occurring in the simulations, this nonlinearity is not significant, and the linear elastic models of the cytoskeletal components are fully acceptable. Neither a possible rearrangement of the cytoskeleton as a consequence of the load acting on the cell during its testing was considered because the time needed for it is longer than the typical time of an experiment (e.g., 5 up to 10 minutes for rearrangement of microtubules); therefore, these processes cannot manifest during this time. Also, the nonlinear behaviour of integrin in focal adhesions [63] is not considered because focal adhesions are represented only by the nodes of the bendotensegrity structure in our model. Although the number of cytoskeletal elements is significantly lower than in a real cell, it was shown that this number is not decisive for the quality of the model [27, 30, 43, 57], and the authors do not know of any discrete model having the number of elements comparable with reality.

## 5. Conclusion

The FE bendotensegrity models of endothelial cells with different shapes were used for simulations of different mechanical loading conditions. Some of them were validated using experimental results in the literature. The model with the shape corresponding to real cell geometry within an arterial wall was loaded by loads corresponding to those induced by a physiological blood flow. In the investigated models, the impact of different loads on individual cell components was evaluated and the role of individual cytoskeleton components was assessed. It was shown that in cell stiffness, the AFs play the dominating role, with a significant contribution of MTs under high tensile loads. Principal strains in the nucleus are hypothesized as quantities decisive for mechanotransduction, and the presented models enable comparing them under different loading conditions. In the future, the model can be expanded to a cell population in the endothelium layer and combined with corresponding biological experiments quantifying the biological response of the cells. Thus, we could investigate the impact of different loading conditions in the arterial wall on remodelling or disruption of the endothelium layer which is decisive in the initial phase of atherosclerosis.

## Figures and Tables

**Figure 1:** Arrangement of cytoskeletal components with respect to the nucleus in the flat and dome models (a); continuous elements of the flat model (b); front view of the dome model (c).

**Figure 2:** Suspended cell model for simulation of the compression test: (a) unloaded cytoskeleton in front view and (b) unloaded model in wire frame and under 50% compression.

**Figure 3:** Suspended cell model for consecutive steps in simulation of tensile test: (a) unloaded spherical cell, (b) compressing the cell by 20%, and (c) stretching the cell by 50%.

**Figure 4:** Structural arrangement of cytoskeletal components with respect to the nucleus in the adherent cell model.

**Figure 5:** Adherent cell model in simulation of compression test at its initial shape and under 50% compression (blue).

**Figure 6:** Comparison of simulations of suspended cell compression with force-deformation curves from the corresponding experiments in [47, 53]. The highest, medium, and lowest stiffness curves are taken from the experimental results.

**Figure 7:** Comparison of the simulated force-deformation curve in tension with the experimental response obtained with cultured bovine aortic endothelial cells [49].

**Figure 8:** Comparison of simulated force-deformation curves obtained with the adherent cell and flat cell models with the experimental curves from [47]. The highest, medium, and lowest stiffness curves are taken from the experimental results.

**Figure 9:** Simulation results of 50% cell compression: stresses in (a) AFs (isometric view), (b) IFs (top view), and (c) MTs (isometric view); (d) distribution of first principal (logarithmic) strain in the nucleus.

**Figure 10:** Simulation results of 50% elongation of a suspended cell: axial stress distribution in (a) AFs, (b) IFs, and (c) MTs; (d) distribution of first principal (logarithmic) strain in the nucleus.

**Figure 11:** Distribution of (a) the first and (b) third (maximal negative) principal (logarithmic) strains in the nucleus of an adherent endothelial cell under 50% compression.

**Figure 12:** Distribution of (a) the first and (b) third (maximal negative) principal (logarithmic) strains in the nucleus of the flat endothelial cell model under 50% compression (isometric view).

**Figure 13:** Distribution of first principal strain in the nucleus of flat- (a) and dome-shaped (b) endothelial cell models under 1.87 Pa shear stress.

**Figure 14:** Distribution of shear strain in the cytoplasm of the flat- (a) and dome-shaped (b) models of endothelial cells under 1.87 Pa shear stress.

**Figure 15:** Contribution of cytoskeletal components in a spherical cell model to its stiffness (a) in compression and (b) in tension. The reaction force is normalized to 1 with respect to that from the hybrid model.

**Figure 16:** Contribution of cytoskeletal components in cell models to their stiffness in compression: (a) adherent model; (b) flat model. The reaction force is normalized to 1 with respect to that from hybrid model.

**Table 1:** Finite elements used for discrete components of the cell models and their elastic parameters.

Cell component	Elastic modulus, *E* (Pa)	Poisson's ratio, *υ*	Diameter (nm)	Finite element specification	Nature
Microtubules (MTs) [45]	1.2 × 10^9^	0.3	25/17 (outer/inner)	BEAM188	Curved beams
Actin filaments (AFs) [46]	2.2 × 10^9^	0.3	4.5	LINK180	Tension only trusses
Intermediate filaments (IFs) [46]	2.0 × 10^9^	0.3	10	LINK180	Tension only trusses
Actin bundles (ABs) [41]	0.34 × 10^6^	0.3	250	LINK180	Tension only trusses

**Table 2:** Finite elements used for continuous components of the cell models and their hyperelastic parameters.

Component name	Young's modulus, *E* (Pa)	Shear modulus, *G* (Pa)	Bulk modulus, *K* (Pa)	Finite element specifications
Cytoplasm [47]	0.5 × 10^3^	0.17 × 10^3^	2.77 × 10^3^	Solid 185
Nucleus [47]	5 × 10^3^	1.7 × 10^3^	27.77 × 10^3^	Solid 185
Cell membrane (CM) [31]	1 × 10^6^	0.33 × 10^6^	Infinity	Shell 181
Actin cortex (AC) [48]	2 × 10^3^	0.67 × 10^3^	Infinity	Shell 181

## Data Availability

The data sets generated and analysed during the current study are available from the corresponding author upon request.
